# Early Family Intervention in Children with Language Delay: The Effect of Language Level and Communication Ability

**DOI:** 10.1155/2022/3549912

**Published:** 2022-05-13

**Authors:** Bo Zhao, Yu Liu, Jing Liu, Yurui Liu

**Affiliations:** ^1^Child Healthcare Department, The Third Affiliated Hospital of Zunyi Medical University (The First People's Hospital of Zunyi), Zunyi 563000, China; ^2^Child Healthcare Department, Maternal and Child Health Hospital of Zigong, Zigong, China

## Abstract

Language development delay refers to the children's oral expression ability or language understanding ability obviously lagging behind the normal development level of children of the same age. The efficacy of early family intervention in children with language delays is promising. The observational study was conducted involving 120 children aged 0∼3 years treated in the pediatric health department of the Third Affiliated Hospital of Zunyi Medical University for language delay. They were assessed for eligibility and recruited. The eligible children were grouped by 1 year, 2 years, and 3 years and were assessed on the Gesell Developmental Schedules and Normal Development of Social Skills from Infant to Junior High School Children (S-M) at the time of initial diagnosis and after the family language intervention. The family language intervention was performed by the parents and lasted for 6 months. All eligible children had a development quotient (DQ) > 86 in motor ability before and after the intervention. All eligible children had a DQ < 86 before the family language intervention in adaptive ability, social ability, and language ability and a DQ > 86 after the intervention. Family language intervention was associated with significant improvement in social life skills in all children, with higher independent living, exercise, operation, interaction, and participation in group activities and self-management after the intervention. Early family intervention yields significant efficacy in children with language delays in Zunyi City by improving the language ability and communication ability of young children, which provides a reference for clinical treatment.

## 1. Introduction

Language delay is a common developmental issue in children [1], which refers to language development that follows the normal developmental sequence but lags behind the normal development [2]. Its incidence is about 15%, and children aged 18 to 35 months with only language delays were defined as “late talkers” [3]. Zhang et al. [4] proposed that children aged 2 to 3 years with a vocabulary of less than 30 words at 24 months and less than 3/5 structural expressions at 30 months for boys/girls are considered delayed in language development [5]. Children with language delays lag behind their normal peers in vocabulary development, sentence length, tone changes, and reading ability and experience verbal and interpersonal communication issues as well as cognitive, literacy, numeracy, and behavioral difficulties [6]. Currently, language skills assessments are mostly performed using the Gesell Developmental Schedules, in which a verbal ability with a DQ < 86 is defined as language delays. A low score on the language assessment at the initial diagnosis of a child with language delays is associated with a high level of severity and poor prognosis [7]. The prolonged duration of language delays and delayed diagnosis may result in severe deficits and issues other than mere language problems [8]. Early detection and intervention for language developmental abnormalities may achieve a significant reduction in the short- and long-term adverse effects on children. The development of children before the age of 3 heavily relies on the parenting style [9]. This period is a critical time for children's language development, and language interventions at this stage facilitate the prevention of negative effects due to language disorders [10]. With the guidance of a language therapist, parents can gain a more accurate understanding of their children's language skills and help them adapt to the therapeutic environment (the treatment environment is altered from the hospital to the child's living environment) [11]. Research related to language delays has become a hot spot in developmental behavior pediatric research in China in recent years [12]. However, the Gesell assessment requires qualified professionals to ensure the accuracy of the assessment, which demands quality training for family intervention practitioners.

Accordingly, this paper puts forward the concept of “family early intervention,” which is “a series of activities such as education, rehabilitation training, nutrition, and health care for preschool children with developmental disorders or possible disorders within the family” to provide early family intervention for children with autism and promote their physical, psychological, and social adaptation [13].

The aim of this study was to study the effect of early family intervention on children with language delays. The results are reported as follows.

## 2. Materials and Methods

### 2.1. Research Subjects

The observational study was conducted involving 120 children aged 0∼3 years treated in the pediatric health department of the Third Affiliated Hospital of Zunyi Medical University for language delay. They were assessed for eligibility and recruited. The eligible children were grouped by 1 year, 2 years, and 3 years and were assessed on the Gesell Developmental Schedules and Normal Development of Social Skills from Infant to Junior High School Children (S-M) at the time of initial diagnosis and after the family language intervention. The protocol of the study was ethically approved by the Ethics Committee of the Zunyi Medical University (2018-3398/23).

### 2.2. Inclusion and Exclusion Criteria

#### 2.2.1. Inclusion Criteria

The language abilities DQ of the Gesell Developmental Schedules was <86 [14].

#### 2.2.2. Exclusion Criteria

(1) With autism; (2) with severe heart, liver, and kidney function diseases, and neurological disorders; (3) with hearing impairment.

### 2.3. Methods

The Gesell Developmental Schedules and Normal Development of Social Skills from Infant to Junior High School Children (S-M) assessments were performed for each child at the initial visit (The Gesell assessment kits are available in out department, with qualified professional staff and resources to allow the realization of this study). Simple and compound language delays were defined as per Gesell Developmental Schedules, with hearing impairment excluded, and grouped by age 1, 2, and 3 years. The parents were first trained to provide instructional assistance to the children, including vocal and verbal stimulation during play, breastfeeding, oral function training, and other skills training, and they were instructed to speak aloud to the children with exaggerated facial expressions, respond positively to their needs and voices, and abstain from electronic media, followed by a 6-month home language intervention therapy performed by the parents. The Gesell Developmental Schedules and Normal Development of Social Skills from Infant to Junior High School Children (S-M) assessment was performed again after the treatment.

### 2.4. Outcome Measures

1. Hearing impairment: hearing impairment was excluded by aberration product evoked otoacoustic emissions (OAE) combined with behavioral audiometry.
2. Compound issues: the DQ values of the four domains of the Gesell Developmental Schedules were used to define the issues. A mere language DQ < 86 was considered simple language delays. A language DQ < 86 with more than one of the motor, adaptive, or social DQs <86 was considered compound issues.
3. Gesell Developmental Schedules: the test is administered to children from birth to 5 years of age, with emphasis on those under 3 years of age. The test lasts about 30 minutes and focuses on the four areas of motor, adaptive, language, and social abilities. Pass items were marked as “+”, fail items were marked as “−,” those exceeding the requirements were marked as “++” or “++++,” items that showed no response were recorded as “?,” and all data were analyzed to assess intelligence. DQ of the four areas = the measured age/experimental age × 100, and a developmental quotient of <86 indicates language delays.
4. Infant to Junior High School Children (S-M): this scale is used to assess the adaptive behavior of infant to junior high school students, with 132 items. With one point for each item passed, six items of independent living, exercise, operation, interaction, participation in group activities, and self-management were evaluated to understand children's social life ability. The lower the score, the lower the ability of the matching item.

### 2.5. Statistical Analysis

SPSS22.0 software was used for data analyses. The count data were expressed as (*n* (%)) and subjected to the chi-square test. The measurement data were expressed as (*x*− ± *s*) and subjected to the *t*-test. Differences were considered statistically significant at *P* < 0.05.

## 3. Results

### 3.1. General Information

There were 38 cases in the 1-year group, 21 boys and 17 girls, 22 cases of simple language delays, and 16 cases of compound language delays. There were 45 cases in the 2-year group, 22 boys and 23 girls, 26 cases of simple language delays, and 19 cases of compound language delays. There were 37 cases in the 2-year group, 18 boys and 19 girls, 24 cases of simple language delays, and 13 cases of compound language delays (see Table 1).

### 3.2. Gesell Assessments in All Enrolled Children

Early family intervention resulted in significantly higher Gesell assessment results of motor ability, adaptive ability, response ability, and language ability (98.34 ± 18.75, 77.91 ± 12.93, 76.10 ± 11.71, 65.14 ± 9.85) as compared to the results before treatment (104.09 ± 12.93, 91.50 ± 18.82, 98.28 ± 19.32, and 94.89 ± 18.51) of all enrolled children, as shown in Table 2. Before treatment, the Motor ability was 98.34 ± 18.75, the adaptive ability was 77.91 ± 12.93, the response ability was 76.10 ± 11.71, and the language ability was 65.14 ± 9.85. After treatment, the above indicators were 104.09 ± 12.93, 91.50 ± 18.82, 98.28 ± 19.32, and 94.89 ± 18.51, all higher than before (*P* < 0.05).

### 3.3. Gesell Assessments in 0-1-Year-Old Children

The Gesell assessment results of 0∼1-years-olds are shown in Table 3. The children of 0∼1 year showed significantly elevated motor ability, adaptive ability, response ability, and language ability scores (97.87 ± 18.28, 77.88 ± 13.25, 75.84 ± 11.23, 64.83 ± 10.01) than before treatment (103.87 ± 12.99, 91.08 ± 19.23, 97.68 ± 20.02, and 94.68 ± 18.76) (*P* < 0.05).

### 3.4. Gesell Assessments in 1-2-Year-Old Children

The Gesell assessment results of 1-2-year-olds are shown in Table 4. The children of 1∼2 years showed significantly elevated motor ability, adaptive ability, response ability, and language ability scores (98.27 ± 19.33, 77.92 ± 13.01, 76.02 ± 12.01, 65.21 ± 9.83) than before treatment (104.17 ± 13.21, 91.74 ± 18.74, 98.23 ± 18.97, and 94.94 ± 18.35) (*P* < 0.05).

### 3.5. Gesell Assessments in 2-3-Year-Old Children

The Gesell assessment results of 2-3-years-olds are shown in Table 5. The children of 2∼3 years showed significantly elevated motor ability, adaptive ability, response ability, and language ability scores (98.92 ± 19.01, 77.94 ± 12.87, 76.48 ± 12.13, 65.37 ± 9.98) than before treatment (104.21 ± 12.87, 91.65 ± 19.02, 98.96 ± 19.52, and 95.03 ± 18.95) (*P* < 0.05).

### 3.6. Social Life Skills

All eligible children showed significant improvements in social life skills after the intervention, in terms of independent living, motor, operation, interaction, participation in group activities, and self-management (all *P* < 0.05) (Tables 6∼9).

## 4. Discussion

The early developmental stages of children are from birth to adolescence, with the most critical and rapid developmental period being from 0 to 3 years of age, which is highly susceptible to the influence of external factors [15]. Language is a significant ability in children's learning, personality development, and social interactions. Delayed language development compromises the children's social interactions and hinders the development of their social adaptation skills, which is detrimental to their overall development. Family language intervention in the early stages of child development may lower the risk of language disorders, and through scientific guidance, it allows a healthy physical, mental, physical, and cognitive state of the children [16]. With the guidance of a language therapist, parents can obtain a more accurate understanding of their child's language skills and adapt the therapeutic environment for them [17].

Results in the present study showed significant mitigation of language delays in all eligible children. The developmental age of language abilities showed the fastest growth and a clear catch-up effect. This intervention allows increased parent-child communication and interaction to significantly improve the child's ability of environmental adaptation and communication willingness. The response ability also showed a significant improvement, with the intervened children being able to reach normal developmental levels, indicating the effectiveness of early family intervention for children with language delays. Moreover, the results of this study presented significantly enhanced social life skills of the children. Previous research pointed out that the social life skills of children with language delays, including independent living, exercise, interaction, group activities, and self-management skills, are significantly lower than those of normal children, which is consistent with the results of the present study [18]. The reasons for this may be attributed to the poor awareness of the hazards, the late start of diagnosis and intervention of language problems, and the lack of professional language rehabilitation personnel and intervention agencies. Other possible issues include lack of effective communication in family education, excessive family intervention, lack of control over children's behavior, and overprotection or rude scolding. A study by Luo et al. found that parents' love and affection for the fetus during fetal education contributes to the reduction of preschool problems, emphasizing a strong impact of family education on children's behavioral problems [19]. In the present study, parents were trained by pediatric health care practitioners to provide language interventions for children, which is of great significance in improving the social lives of children with language delays. It has been reported that early intervention is effective in improving vocabulary and overall phonological development, and in addition to language-related progress, it also improves the child's social skills, increases self-confidence, and relieves parental stress, resulting in better language progress, which remains consistent with the results of the present study [20]. However, this paper still has the following limitations. This study was an observational study without a control group. In addition, the number of children included in this study was small and the follow-up time was short, which failed to explain the long-term impact on children. Large sample, multicenter, long follow-up randomized controlled studies will be conducted in the future.

## 5. Conclusion

Early family intervention yields significant efficacy in children with language delays in Zunyi City by improving the language level and communication ability of young children, which provides a reference for clinical treatment.

## Figures and Tables

**Table 1:** Baseline data of research subjects (%).

	Total (*n* = 120)	0∼1 year (*n* = 38)	1∼2 years (*n* = 45)	2∼3 years (*n* = 37)
Gender				
Male	61	21	22	18
Female	59	17	23	19
Language delays types				
Simple	72	22	26	24
Compound	48	16	19	13

**Table 2:** Gesell assessments results of all enrolled children.

	Before intervention	After intervention	*t*	*P*
Motor ability	98.34 ± 18.75	104.09 ± 12.93	2.766	0.006
Adaptive ability	77.91 ± 12.93	91.50 ± 18.82	6.52	<0.001
Response ability	76.10 ± 11.71	98.28 ± 19.32	10.75	<0.001
Language ability	65.14 ± 9.85	94.89 ± 18.51	15.54	<0.001

**Table 3:** Gesell assessments results of 0-1-year-old children.

	Before intervention	After intervention	*t*	*P*
Motor ability	97.87 ± 18.28	103.87 ± 12.99	1.649	0.103
Adaptive ability	77.88 ± 13.25	91.08 ± 19.23	9.484	0.001
Response ability	75.84 ± 11.23	97.68 ± 20.02	58.65	<0.001
Language ability	64.83 ± 10.01	94.68 ± 18.76	8.654	<0.001

**Table 4:** Gesell assessments results of 1-2-year-old children.

	Before intervention	After intervention	*t*	*P*
Motor ability	98.27 ± 19.33	104.17 ± 13.21	1.690	0.095
Adaptive ability	77.92 ± 13.01	91.74 ± 18.74	4.064	<0.001
Response ability	76.02 ± 12.01	98.23 ± 18.97	6.636	<0.001
Language ability	65.21 ± 9.83	94.94 ± 18.35	9.580	<0.001

**Table 5:** Gesell assessments results of 2-3-year-old children.

	Before intervention	After intervention	*t*	*P*
Motor ability	98.92 ± 19.01	104.21 ± 12.87	1.402	0.165
Adaptive ability	77.94 ± 12.87	91.65 ± 19.02	3.631	0.001
Response ability	76.48 ± 12.13	98.96 ± 19.52	5.950	<0.001
Language ability	65.37 ± 9.98	95.03 ± 18.95	8.424	<0.001

**Table 6:** Social life skills of all enrolled children.

	Before intervention	After intervention	*t*	*P*
Independent living	9.80 ± 0.61	10.14 ± 0.56	4.498	<0.001
Motor	9.50 ± 0.92	10.03 ± 0.44	5.693	<0.001
Operation	9.63 ± 0.95	10.29 ± 0.60	6.435	<0.001
Interaction	9.69 ± 0.80	10.12 ± 0.47	5.077	<0.001
Participation in group activities	9.33 ± 1.00	10.12 ± 0.51	7.709	<0.001
Self-management	8.49 ± 1.61	10.15 ± 0.66	10.45	<0.001

**Table 7:** Social life skills of 0-1-year-old children.

	Before intervention	After intervention	*t*	*P*
Independent living	9.78 ± 0.62	10.01 ± 0.34	2.005	0.049
Motor	9.21 ± 0.87	9.98 ± 0.47	4.800	<0.001
Operation	9.37 ± 0.95	10.27 ± 0.64	4.843	<0.001
Interaction	9.53 ± 0.85	10.08 ± 0.42	3.576	<0.001
Participation in group activities	9.21 ± 0.98	10.02 ± 0.53	4.482	<0.001
Self-management	8.01 ± 1.25	9.99 ± 0.87	8.014	<0.001

**Table 8:** Social life skills of 1-2-year-old children.

	Before intervention	After intervention	*t*	*P*
Independent living	9.80 ± 0.59	10.18 ± 0.65	2.904	0.005
Motor	9.55 ± 0.91	10.05 ± 0.42	3.347	0.001
Operation	9.56 ± 0.84	10.26 ± 0.68	4.345	<0.001
Interaction	9.69 ± 0.74	10.13 ± 0.51	3.284	<0.001
Participation in group activities	9.32 ± 1.03	10.15 ± 0.52	4.826	<0.001
Self-management	8.52 ± 1.65	10.17 ± 0.59	6.317	<0.001

**Table 9:** Social life skills of 2-3-year-old children.

	Before intervention	After intervention	*t*	*P*
Independent living	9.81 ± 0.64	10.21 ± 0.62	2.731	0.008
Motor	9.73 ± 0.94	10.07 ± 0.43	2.001	0.049
Operation	9.98 ± 1.02	10.35 ± 0.44	2.026	0.046
Interaction	9.82 ± 0.81	10.14 ± 0.49	2.056	0.043
Participation in group activities	9.46 ± 1.01	10.18 ± 0.47	3.931	<0.001
Self-management	8.94 ± 1.79	10.29 ± 0.41	4.472	<0.001

## Data Availability

All data generated or analyzed during this study are included in this published article.
